# Extremely Reduced Motion in Front of Screens: Investigating Real-World Physical Activity of Adolescents by Accelerometry and Electronic Diary

**DOI:** 10.1371/journal.pone.0126722

**Published:** 2015-05-08

**Authors:** Judith Streb, Thomas Kammer, Manfred Spitzer, Katrin Hille

**Affiliations:** 1 ZNL Transfercenter of Neuroscience and Learning, University of Ulm, Ulm, Germany; 2 Department of Psychiatry, University of Ulm, Ulm, Germany; Vanderbilt University, UNITED STATES

## Abstract

This paper reports accelerometer and electronic dairy data on typical daily activities of 139 school students from grade six and nine. Recordings covered a typical school day for each student and lasted on average for 23 h. Screen activities (watching television and using the computer) are compared to several other activities performed while sitting (e.g., playing, eating, sitting in school, and doing homework). Body movement was continuously recorded by four accelerometers and transformed into a motion sore. Our results show that extremely low motion scores, as if subjects were freezing, emerge to a greater extent in front of screens compared to other investigated activities. Given the substantial amount of time young people spend in front of screens and the rising obesity epidemic, our data suggest a mechanism for the association of screen time and obesity.

## Introduction

Blank stares and sitting absolutely motionless − that’s the impression many parents get when they see their children watching television. This almost complete absence of motion (i.e., “freezing”) is not observed in other sedentary behavior, such as sitting at the dinner table or in class. Although an association between television viewing and decreased physical activity seems to be common knowledge, it has received little scientific attention. To our knowledge, only two studies specifically address freezing in front of television: DuRant et al. [1] measured the activity level of each minute of the day by observation using the Children’s Activity Rating Scale. Their results showed that physical activity was lower during television watching than during no television watching. Dietz et al. [2] examined the movement effects of television viewing, reading, and sitting quietly for 15 minutes in a laboratory setting. Physical activity was assessed in two ways: By using four Caltrac monitors taped to the hands and feet and by a observational count of movements observed on a videotape. The objective measured activities via Caltrac monitors did not differ significantly between the three conditions, whereas observed movements were found to be significantly increased when the children were sitting than when they were reading or watching television.

Additional studies [3–9] investigated children’s daily physical activity and their amount of watching television. But none of them did investigate specifically decreased movements while watching TV. Most of them compared the average duration of watching television (usually assessed by a questionnaire) and the overall daily physical activity (usually assessed by accelerometry). To sum up, up to now, there is no objective evidence confirming the impression that sitting in front of a television or computer screen causes freezing behaviour.

The present study combines the pros of the two studies mentioned above: We utilized the most reliable method for investigating real-world physical activity − 24 hour accelerometer monitoring during a normal day. Dietz et al. [2] fixed their sensors solely to the hands and feet, measuring the amount of fidgeting with arms and legs. Unlike Dietz et al. [2] we fixed a tri-axial acceleration sensor to the torso (i.e., at the sternum) and a uni-axial sensor to the right thigh in order to assess gross movements of the torso and the more fidgeting movements of the limbs. Data from 139 school students were recorded and more than 3,000 hours were analyzed. The accelerometer data were summarized and median motion scores were computed for several daily activities of the students. These were assessed using a handheld PC which prompted the students to briefly respond to a quick activity questionnaire at regular intervals.

## Materials and Methods

### Subjects

Subjects were recruited in schools after the headmasters and teachers agreed to take part with their school in the study (note: recording took place during lessons, too). Students and their parents were informed through a letter and in an informative meeting as part of parents’ evenings at school. The study was explained in the letter and at the meeting. Questions about the study were answered in the meeting or by phone. Participation was voluntarily. All students were eligible to take part as long as they had no severe chronic diseases like epilepsy or cardiac defects. Students were given a specific date for their participation, according to a predefined scheme. There were very few requests to change these dates e.g. when the recording day fell on a day when the participant wanted to train for swimming championships. 143 students volunteered for participation after an informative meeting and were given shopping vouchers for taking part. Their parents signed an informed consent statement. Data of four subjects had to be discarded because of missing data from the handheld PC due to recording artifacts. Thus, data of 139 students (68 boys) were analyzed. The sample included 77 sixth graders (42 boys; mean age = 11) and 62 ninth graders (29 boys, mean age = 15). The study was approved by the institutional review board of the University of Ulm.

### Motion recording and processing

Accelerometry was carried out with a general purpose digital recorder designed for prolonged ambulatory recording (Varioport, Becker Meditec, Karlsruhe, Germany). The physical activity was measured by two accelerometers: a tri-axial and a uni-axial sensor. The first sensor was placed at the sternum, the sensitive axes pointing in the longitudinal, sagittal, and transversal directions. The second sensor was placed in the middle of the right thigh. The motion sensors directly measured acceleration of earth gravity in milli-g (~cm/s^2^). The motion signal was recorded with low pass filtering at 10 Hz and a sampling rate of 32-Hz. An acceleration index called the motion score (MS) was computed as follows: The raw signal of the activity channels (sternum longitudinal, sagittal, and transversal and thigh sagittal) was high pass filtered (cut off frequency 0.1 Hz, 3dB). Then, the dynamic signal of the 4 accelerometers was summed up: s = sqrt(a_1_^2^ + a_2_^2^ + a_3_^2^ + a_4_^2^). Finally, MS was calculated by the linear transformation: MS = 129.99 + 43.361*log(s). This transformation yielded a MS value of 0 with a motion of about 0.05 g, MS 100 with 0.5 g, MS 200 with 5 g, etc. (see [10]). The distributions of the motion scores for the subjects were positively skewed with many incidents of little movement and a decreasing amount of incidents of more movement including outliers. As the median is less sensitive to these outliers than the mean we opted for median motion scores rather than mean motion scores.

### Electronic diary

A handheld computer was given to the student as an electronic diary. A vibration alarm was generated by the Varioport recorder every 15 ± 4 minutes, i.e., the alarm was generated on average every 15 minutes, with a minimal time window of 11 and a maximal time window of 19 minutes. This alarm signaled the students to answer a set of predefined questions on their handheld computer. The subjects were asked to provide the following information for the minute immediately prior to the alarm: body posture (lying, sitting, standing, walking, running/sport/bicycle) and present location (at school, at home, elsewhere, en route). If the students stated to be at school, they were requested to specify the lesson. If they stated to be at home or elsewhere, they were asked to select their current activity (e.g. watching television, playing, homework, eating). This scheme worked quite well for categorizing students’ activities, as the category “other” was selected as primary activity in only 13.5% of all entries. Students contributed an average of 54 entries per day in the electronic diary (SD = 11.5, range 24 to 73). We computed the “compliance rate” by dividing the number of entries received by the number of entries requested during a student’s day time. For example, if a participant had completed 40 entries at the 50^th^ request, that participant’s compliance rate was 80%. The mean compliance rate was 94% (SD = 5.7; range 70 to 100). Data from the handheld computer and the Varioport recorder were synchronized and merged.

### Procedure

Each student was equipped with the ambulatory monitoring system during one regular school day. The acceleration sensors and the Varioport recorder were attached to the student at school before the lessons began. When going to bed students were requested to turn off the vibration alarm in order to avoid getting awakened by the prompt. The students were monitored for almost a full day. At the next day before school the acceleration sensors and the Varioport were taken off. The average recording time was 22 h 38 min (Min 11 h 19 min, Max 24 h 51 min) per student—adding up to over 3,000 hours of motion recording.

### Statistical analysis

The median motion score for the activities logged by the electronic diary was computed from the accelerometer data separately for each subject. A Friedman test was calculated with the dependent variable “median motion score” and the repeated measurement factor “activity”. The latter comprised the following activities performed while sitting: attending classes, doing homework, watching television and using a computer. Subordinate analyses (Wilcoxon pairwise comparisons) were computed if the Friedman test revealed significant results.

In addition, for each of the four activities (attending classes, doing homework, watching television and using a computer—all performed while sitting) and for each subject the motion scores (units per minute) were grouped according to the following categories: scores between 0 and 5, 5 and 10, 10 and 15, 15 and 20, 20 to 25 and all above 25. Scores between 0 and 5 correspond to extremely reduced motion, i.e., for an observer, students have sat absolutely motionless. Mean percentages were calculated separately for each activity. For the lowest motion score category (0–5) a Friedman test and subordinate analyses (Wilcoxon pairwise comparisons) were carried out.

## Results

As can be seen in Fig 1, among activities that were performed while sitting, we found extremely low median motion scores (±interquartile range) for screen activities, i.e. watching television (8.8 ± 14.7; n = 114) and using a computer (11.2 ± 17.4; n = 73). In comparison, the scores of some other sedentary daily activities were substantially higher: playing (41.6 ± 32.7; n = 47), talking (30.8 ± 30.8; n = 99), eating (26.9 ± 25.7; n = 130), attending classes (20.6 ± 11.7; n = 139) and doing homework (19.4 ± 17.9; n = 97). For a within-subject analysis, we included only those students who engaged in each of the following sedentary activities during their monitoring day: attending classes, doing homework, watching television, and using a computer (n = 33). Friedman’s ANOVA revealed significant differences between median motion scores of these activities (Chi^2^(3) = 18.1, P<0.001) that could be attributed to the differences between screen- and non-screen-activities (see Table 1).

**Fig 1:** Mean physical activity assessed during each activity, quantified as motion score (MS), i.e. log(vector sum of acceleration), see Methods. Zero represents almost null physical activity (0.05g), 60 represents a very high activity level (0.2 g). The vertical line indicates the median of physical activity across all subjects. Bubble area indicates the percentage of subjects performing the labeled activity. The largest bubble (“attending classes” corresponds to 100% of the subjects, and the smallest bubble (“creative work”) corresponds to 9% of the subject. Bubbles are distributed along the y-axis for sake of clarity.

**Table 1:** Wilcoxon pairwise comparisons between four sedentary behaviors: Doing homework, attending classes, using a computer and watching television.

	Homework vs. Class	Television vs. Computer	Television vs. Homework	Computer vs. Homework	Television vs. Class	Computer vs. Class
Z	-.223	-1.474	-2.582	-2.082	-3.261	-2.350
P-Value	.823	.140	.010	.037	.001	.019
Cohen’s d	.09	.03	.66	.33	.83	.35

The second analysis shows that extremely low motion scores were found to a significant greater extent during sitting in front of screens as compared to sitting while doing other things [Friedman’s ANOVA for proportion of minutes with motion scores between 0–5: Chi^2^(3) = 11.1, P = 0.011; Wilcoxon pairwise comparisons: school lessons vs. television (P<.001) resp. computer (P<.001); homework vs. television (P = .030)]. Fig 2 illustrates this effect: About 30% of the time spent in front of screens is accompanied by extremely low motion scores (motion scores between 0 and 5).

**Fig 2:** Proportion of minutes sorted by (the height of the) motion score for different activities (attending classes, doing homework, watching television and using a computer). Low motion scores (0–5) indicate little physical activity in the minute recorded. High motion scores were summarized in a large cluster (26–121) as this was not the focus of this study.

## Discussion

Students sit in class, they sit while doing homework, while commuting, and at mealtimes. In recent years, student life became ever more sedentary as they spend a substantial part of their leisure time sitting in front of screen media. While all these activities involve sitting, our analyses suggest that there are behavioral differences regarding the amount of physical motion while sitting: If students sit in front of screens, they become extremely motionless.

The main objective of the study was to compare several kinds of daily activities with regard to their motion scores. Different activities go together with different motion scores. On a descriptive level across all subjects: The lowest level of activity was recorded while students were watching television or using a computer. No other daily activities—even sedentary ones such as reading—were accompanied by an absence of physical movements as large as was observed during sitting in front of a screen.

Motion scores differed not only between activities but also between subjects. Therefore, comparing activities requires a within subject design. The sample of 33 students did not only visit school and did homework but also chose to watch TV and to use a computer on the day of recording. All these activities were performed while sitting and classified as sedentary. From the data, it appeared that not all forms of sitting are equal in terms of body movements: When subjects sat in front of screens they showed even lower motions scores compared to sitting in class or while doing homework; they appeared to be completely motionless in front of the screens. This was confirmed by our analyses focusing very low activity counts. The issue has been discussed by others [1–3], but this study is the first to provide evidence by direct measurement.

Dietz et al. [2] detected significant differences in physical activity measured during screen time compared to other sedentary behavior by fixing sensors to the hands and feet. We fixed our sensors to the torso. So even excluding movements with arms and legs as a main source of movement while sitting, TV- and computer-screens reduce gross physical motion to a larger extent than sitting while engaged in other activities.

The results could support a mechanism for the link between screen time and obesity which has been suggested by Levine and coworkers [11]: Non-exercise activity thermogenesis (NEAT) is the most variable component of energy expenditure, ranging from 15% of the total energy expenditure in very sedentary individuals, to 50% or more of total energy expenditure in highly active individuals. NEAT is the energy expended for everything that is not sleeping, eating, or sports-like exercises. It includes the energy expended for *changes in posture* and movement during the routines of daily life (e.g., fidgeting, walking, typing, performing yard work). According to the data of our study, NEAT is reduced in front of screens because body posture readjustments are highly reduced.

Our results are consistent with those who correlate TV time with obesity [4]. Most of them have focused on increasing physical activity and decreasing sedentary behavior when trying to reduce obesity.

It must be noted, however, that our study is only correlational in nature thereby ruling out causal conclusions. It might be argued that a very low level of energetic arousal could cause subjects to choose watching television or using computers.

Our study describes and quantifies the effect of extremely reduced motion in front of screens, but it cannot offer a psychophysiological explanation. Different explanations seem possible: (1) The content of screen media is designed to grab and hold the attention of the viewer. It might be that the viewers’ high level of attention renders them motionless. Possibly, the viewers are overwhelmed in an attempt to follow the content, which renders them motionless. (2) Extremely reduced motion has been found to accompany anxiety and fear reactions. From our study, we cannot answer the question of whether such “freezing” behavior is the cause of the observations we made. Further studies with measurements of muscle tone in addition to muscle movements are needed to resolve this open question.

Given the amount of time children and adolescents spend in front of screens as well as the epidemic proportion of obesity in this age range, our results are of importance for general health and the prevention of major non-communicable disorders.

## Supporting Information

S1 Data Data on Motion Score for subjects and their activities (e.g. attending classes, relaxing, eating). (CSV)

S2 Data Data on Motion Score for subjects per condition (attending classes, doing homework, watching TV, using a computer). (CSV)
